# Review and Analysis of Two Gitelman Syndrome Pedigrees Complicated with Proteinuria or Hashimoto's Thyroiditis Caused by Compound Heterozygous *SLC12A3* Mutations

**DOI:** 10.1155/2021/9973161

**Published:** 2021-05-10

**Authors:** Jian-hui Zhang, Dan-dan Ruan, Ya-nan Hu, Xing-lin Ruan, Yao-bin Zhu, Xiao Yang, Jia-bin Wu, Xin-fu Lin, Jie-wei Luo, Fa-qiang Tang

**Affiliations:** ^1^Shengli Clinical Medical College of Fujian Medical University, Fuzhou 350001, China; ^2^Fujian Provincial Hospital, Fuzhou 350001, China; ^3^Department of Neurology, Fujian Medical University Union Hospital, Fuzhou 350001, China; ^4^Department of Traditional Chinese Medicine the First Affiliated Hospital, Fujian Medical University, Fuzhou 350001, China; ^5^Teaching and Research Office of Medical Cosmetology, Department of Management, Fujian Health College, Fuzhou 350001, China

## Abstract

Gitelman syndrome (GS) is an autosomal recessive inherited salt-losing renal tubular disease, which is caused by a pathogenic mutation of *SLC12A3* encoding thiazide-sensitive Na-Cl cotransporter, which leads to disturbance of sodium and chlorine reabsorption in renal distal convoluted tubules, resulting in phenotypes such as hypovolemia, renin angiotensin aldosterone system (RAAS) activation, hypokalemia, and metabolic alkalosis. In this study, two GS families with proteinuria or Hashimoto's thyroiditis were analyzed for genetic-phenotypic association. Sanger sequencing revealed that two probands carried *SLC12A3* compound heterozygous mutations, and proband A carried two pathogenic mutations: missense mutation Arg83Gln, splicing mutation, or frameshift mutation NC_000016.10:g.56872655_56872667 (gcggacatttttg>accgaaaatttt) in exon 8. Proband B carries two missense mutations: novel Asp839Val and Arg904Gln. Both probands manifested hypokalemia, hypomagnesemia, hypocalcinuria, metabolic alkalosis, and RAAS activation; in addition, the proband A exhibited decreased urinary chloride, phosphorus, and increased magnesium ions excretion, complicated with Hashimoto's Thyroiditis, while the proband B exhibited enhanced urine sodium excretion and proteinuria. The older sister of proband B with GS also had Hashimoto's thyroiditis. Electron microscopy revealed swelling and vacuolar degeneration of glomerular epithelial cells, diffuse proliferation of mesangial cells and matrix, accompanied by a small amount of low-density electron-dense deposition, and segmental fusion of epithelial cell foot processes in proband B. Light microscopy showed mild mesangial hyperplasia in the focal segment of the glomerulus, hyperplasia, and hypertrophy of juxtaglomerular apparatus cells, mild renal tubulointerstitial lesions, and one glomerular sclerosis. So, long-term hypokalemia of GS can cause kidney damage and may also be susceptible to thyroid disease.

## 1. Introduction

Gitelman syndrome (GS) is an autosomal recessive hereditary salt-losing renal tubular disease. Hillel J. Gitelman reported three familial diseases characterized by hypokalemia, hypomagnesemia, hypochloremic alkalosis, and hypocalciuria in 1966, and the syndrome was named after him [1]. The prevalence of GS is approximately 1-10 per 40000 people, and the prevalence of heterozygotes is about 1% in western countries [2, 3]. However, in Asia, the prevalence of GS has significantly increased to 10.3 per 10000 people [4], and mutations may be as high as 3% [3]. China reports are fewer, and the number of samples in these reports is comparatively small. GS is inherited in an autosomal recessive mode, and its pathogenic gene is the *SLC12A3* gene (MIM:600968; NC_000016.10), which is located on human chromosome 16q13 and consists of 26 independent exons [5]. Currently, a variety of pathogenic mutations have been discovered, including nonsense mutations, missense mutations, frameshift mutations, deletions, insertions, and splice site mutations [6]. The hot spot mutation site is not yet known. In this study, two GS pedigrees with compound heterozygous mutation presenting with proteinuria or Hashimoto's thyroiditis phenotype were reported. We observed damage to renal tissue in the case of *SLC12A3* mutations causing GS through renal biopsy and discussed the possible relationship between GS and renal pathology and thyroid function.

## 2. Materials and Methods

### 2.1. Subjects

The study included 16 cases from 2 GS pedigrees, specifically 3 males and 6 females from Pedigree A and 5 males and 2 females from Pedigree B. Both pedigrees had no consanguineous marriages. Proband II6 (proband A) of Pedigree A, a female, aged 42, married, with a blood pressure of 124/76 mmHg, and a BMI of 21.22 kg/m^2^, was admitted to the hospital with the chief complaint of “repeated fatigue for one year and chest tightness for one month.” The serum potassium checked locally was 2.95 mmol/L, the chest tightness and palpitations occurred one month before admission, and general fatigue was obvious. The mother of proband A had long-term hypokalemia with no relevant clinical manifestations. Proband II3 (proband B) of Pedigree B, a male, aged 31,with a blood pressure of 125/79 mmHg, and a BMI of 21.52 kg/m^2^, was admitted to the hospital because of “repeated fatigue and foamy urine for half a year.” The proband had increased urine foam with no obvious induction half a year before admission, no decrease in urine output, and no swelling on the face or lower limbs. After testing at the local hospital, the serum potassium level was determined to be 2.33 mmol/L, and this level fluctuated from 2.3 to 2.7 mmol/L after oral potassium supplementation. The older sister of proband B had chronic hypokalemia, which mainly manifested as paroxysmal weakness of limbs and muscle spasms. None of the patients had a low potassium diet or complained of long-term vomiting, diarrhea, or other symptoms. They also had no history of overuse of diuretics, laxatives, or alcohol and no history of drug addiction. No other extrarenal and renal causes of hypokalemia, such as Cushing syndrome, primary aldosteronism, reninoma, Liddle syndrome, renal tubular acidosis, diabetic ketoacidosis, and renal artery stenosis, were found, and there was no history of nephrotoxic drugs or licorice intake. This study was approved by the Ethics Committee of Fujian Provincial Hospital, and all family members participating in this study provided signed informed consent.

### 2.2. Detection Methods

Genomic DNA was extracted from peripheral blood. Under the principle of informed consent, peripheral blood samples (2 mL) were extracted from the patient, and DNA was extracted using the centrifugal column method. The DNA extraction kit used was the QIAGEN DNA whole blood extraction kit of the Gene Company (QIAGEN DNA whole blood extraction kit; QIAGEN, Hilden, Germany).

For primer design, the *SLC12A3* gene sequence was obtained from GenBank (NC_000016) (MIM:600968), and 26 pairs of primers were designed using primer premier 5 software to amplify all 26 exons of the *SLC12A3* gene (as shown in Table 1). The primers were synthesized by the Beijing Liuhe Huada GenePolytron Technologies Inc.

For PCR product amplification, the reaction system (30 *μ*L) contained 2.5 *μ*L 10× Ex Taq buffer, 2 *μ*L dNTP (2.5 mM), 3 *μ*L forward primer (3.0 mM), 3 *μ*L reverse primer (3.0 mM), 1 *μ*L DNA template l, 0.2 *μ*L Ex Taq, and 18.3 *μ*L H_2_O. Using the PCR instrument (PTC-200 PCR, BIO-RAD), denaturing was started at 94°C for 5 min, followed by denaturation at 94°C for 40 s (each primer TM value), annealing for 40 s, extension at 72°C for 60 s, 35 times circulation, and then extension at 72°C for 10 min.

The PCR products were purified using the methods described in the operating instructions of EZNA™ Gel Extraction Kit (Omega Company), and the sequencing was performed according to the PCR product standard operating procedure of BigDye Terminator v1.1 kit.

For analysis of the DNA sequencing results, the DNAMAN Version 5.2.2 was used for alignment with normal sequences. When a heterozygous deletion or insertion was suspected, PCR products were connected to the PGEM-T Easy (Promega) vector to select subclones for sequencing [7].

## 3. Results

### 3.1. Clinical Phenotype

Among the 16 cases in the two GS pedigrees, 4 cases, the proband of Pedigree A (II6), her older sister (II5), the proband of Pedigree B (II3), and his older sister (II2), met the clinical diagnostic criteria of GS: chronic persistent hypokalemia (<3.5 mmol/L), hypomagnesemia (<0.7 mmol/L), and hypocalcinuria (urinary calcium/urinary creatinine <0.2 mmol/mmol) [8]. However, the mother (I2) of proband A of Pedigree A had long-term mild hypokalemia (serum potassium ranges from 3.0 to 3.5 mmol/L), but comprehensive biochemical indicators had not been collected, and there was insufficient evidence for GS diagnosis. Both probands showed hypokalemia, hypomagnesemia, hypocalcinuria, metabolic alkalosis, blood renin, and angiotensin activation state, and proband A showed decreased urine chloride and phosphorus with increased magnesium ion excretion and thyroid dysfunction. The thyroid color doppler ultrasound of Proband A indicated mild diffuse enlargement of the thyroid gland with clear boundaries and no space occupation; however, the thyroid peroxidase and TG antibodies were elevated, resulting in a diagnosis of “Hashimoto's thyroiditis.” In addition, the electronic gastroscope showed chronic superficial gastritis, and proton pump inhibitors were administered for treatment. Proband B had increased urine sodium excretion, a positive urine routine protein (++), and a significantly excessive 24 h urine protein level. Both patients had normal blood pressure, weakness and numbness of limbs, and occasional heart palpitations, chest tightness, and discomfort. Proband B also showed proteinuria. The older sister of proband B had chronic hypokalemia, accompanied by thyroid dysfunction and elevated thyroid peroxidase antibodies and TG antibodies. The thyroid color doppler ultrasound indicated mild and diffuse thyroid enlargement, which was similar to the result of proband A, and this also led to a diagnosis of “Hashimoto's thyroiditis” (Figure 1, Table 2).

Pathological electron microscopic examination of a renal biopsy of proband B showed that the glomerular capillary endothelial cells had obvious vacuolar degeneration, evidence of red blood cells in some lumens, no obvious endothelial cell proliferation, and open capillary loops. There was no obvious thickening in the parietal layer of the renal capsule, and the parietal cells showed vacuolar degeneration with no obvious proliferation. There was swelling and vacuolar degeneration in the glomerular visceral epithelial cells, and segmental fusion of epithelial cells foot processes. The glomerular mesangial cells and matrix proliferated, accompanied by a small amount of low-density electron-dense deposition. There showed vacuolar degeneration of the renal tubular epithelial cells with no special changes in the renal interstitium. The basement membrane was not significantly thickened, as the thickness was about 300–400 nm. Light microscopy showed mild mesangial hyperplasia in the focal segment of the glomerulus, hyperplasia and hypertrophy of the juxtaglomerular apparatus, and mild renal tubulointerstitial lesions. Renal tubular epithelial cell degeneration (turbidity), no cast, interstitial edema, a small number of lymphocytes, monocytes, and foam tissue cells were observed. The immunohistochemistry results for IgG, IgM, IgA, C3d, C4d, and C1q were all negative (Figure 1).

### 3.2. *SLC12A3* Gene Mutation

The results of amplification and direct sequencing of *SLC12A3* (NM_001126108.2) indicated that the genes of the two probands contained compound heterozygous mutations. Proband A (II6) and the older sister of proband A (II5) both had 2 suspicious pathogenic mutations, one of which was C.248G>A of exon 1, which causes CGG→CAG changes, and leads to Arg83Gln, where arginine was substituted by glutamine resulting in a missense mutation. The other mutation point was NC_000016.10: g.56872655_56872667 (gcggacatttttg>accgaaaatttt) of exon 8, which is a splice site mutation or frameshift mutation; the mother of proband A (I2), as well as II1, II3, III1, and III2 only carried the mutation NC_000016.10:g.56872655_56872667 (gcggacatttttg>accgaaaatttt) heterozygotes, while II4 only carried the mutation Arg83Gln (Figure 2, Table 3). Proband B (II3) and the older sister (II2) of proband B had two mutation sites, which were: c.2516A>T of exon 21, which caused GAT→GTT, where aspartic acid was replaced by valine, leading to Asp839Val; and c.2711G>A of exon 23 which caused CGG→CAG, and arginine was replaced by glutamine, resulting in Arg904Gln (Figure 3). Between them, Asp839Val was inherited from their father (I1), and Arg904Gln from their mother (I2); in addition, III1 andIII2 carried Asp839Val heterozygous mutation, and III3 carried the Arg904Gln mutation. See Figure 1 and Table 3 for pedigree analysis.

## 4. Discussion

A thiazide-sensitive NaCl cotransporter (NCCT) is the main ion transport system of distal convoluted tubules (DCT); 5–10% of sodium and chloride ions filtered from the glomerulus are reabsorbed in DCT [9]. The *SLC12A3* mutation leads to structural changes and/or dysfunctions of NCCT located in the DCT cortex; the reabsorption of NaCl in the DCT is reduced, and the decrease of sodium reabsorption capacity leads to an excessive exchange of sodium ions through Na+/K+ and Na+/H+ compensatory reabsorption. While excreting a large amount of K+ and H+, the reduction of reabsorption also causes hypovolemia, which promotes the synthesis and secretion of renin. This is accompanied by renal cell hyperplasia and hypertrophy, and the entire renin angiotensin aldosterone system (RAAS) is activated, which was verified by the renal biopsy pathology of proband B in this study. The excessive exchange of Na+/K+ and Na+/H+ eventually leads to hypokalemic alkalosis. At the same time, due to the large outflow of chloride ions, the polarity of the distal renal tubular cells increases, which increases the reabsorption of calcium ions, leading to hypocalciuria. A decrease in sodium ion reabsorption can lead to a related decrease in magnesium ion reabsorption, leading to hypomagnesemia. In short, these mutations can cause structural changes of NCCT that destroy its biological effects, affect its reabsorption ability, and lead to electrolyte disorders.

The clinical phenotypes of GS show great heterogeneity [10], and there is no obvious association between genotype and phenotype. A patient may show no clinical symptoms and diagnosis of hypokalemia may only occur on a routine physical examination. Electrolyte disturbances, increased RAAS activity, and other factors lead to common clinical manifestations of GS, such as weakness and numbness of limbs, paresthesia, muscle spasm, convulsion, halophilic, normal or low blood pressure, palpitation, arrhythmia, proteinuria, and hypokalemic nephropathy [11, 12]. Patients with homozygous or compound heterozygous mutations usually exhibit lower blood pressure, and approximately 2% of hypotension is caused by GS [4]. The phenomenon of hypotension was not found in these two pedigrees, which may be related to individual differences or dietary habits. The Arg904Gln variant of *SLC12A3* may increase the risk of EH (essential hypertension) [13–15], which indicates that the Arg904Gln variant may be a functional gain mutation [14]. The fatigue of GS patients is mainly caused by hypokalemia, which is generally considered to be related to the fluctuation of potassium ion concentration in or out of the cells, possibly due to excessive *β*-sympathetic nerve excitation or inherited mutation resulting in abnormal potassium channel activity [16]. The deficiency of potassium and magnesium prolonged the duration of the action potential of cardiomyocytes, resulting in longer QT intervals in 50% of patients, which led to an increased risk of ventricular arrhythmia. GS patients with long-term ventricular tachycardia have been reported [17]; patients diagnosed with GS need to undergo a resting electrocardiogram, even if the electrocardiogram is normal. A dynamic electrocardiogram and exercise electrocardiogram examination should be arranged to identify hidden risks.GS patients are at high risk of chronic kidney disease (CKD); however, this mechanism is complex and has not been clearly elucidated. Chronic hypokalemia can cause renal injury through tubular vacuolization, cysts, and tubulointerstitial nephritis [18], and the pathological report of proband B in this study confirms these results. Some scholars also believe that the increase in circulating renin, angiotensin II, and aldosterone may be more important factors for renal injury and fibrosis [19]. Therefore, it is necessary to closely monitor the renal function indicators of GS patients in clinical practice to improve the prognosis of patients.

It is interesting to note that proband A and the older sisters of proband B both had thyroid dysfunction. The proband A thyroid function test indicated that the patient had autoimmune thyroid disease (AITD) and subclinical hypothyroidism, while the older sister of proband B had AITD and subclinical hyperthyroidism. This information, combined with the color Doppler ultrasound results, and the elevated thyroid peroxidase and TG antibodies, evoked a diagnosis in both of “Hashimoto's thyroiditis (HT).” In the literature review of 18 cases of AITD combined with GS, 13 cases had toxic diffuse goiter (Graves' disease, GD), 3 cases had HT, 2 cases were positive for the simple AITD antibody, and 1 case was a base deletion mutation; the rest were single base substitutions [20]. In the Japanese GS population, the incidence of thyroid dysfunction is 4.3% [21]. The above studies all indicate that GS is associated with thyroid dysfunction, and the incidence could be higher than expected; however, there is still insufficient data to determine whether AITD is more likely to occur in GS patients than other groups. Although there are sufficient data to suggest that hyperthyroidism can lead to hypokalemia and hypomagnesemia, there is still a lack of research on the long-term effects of these on thyroid function, although iodine metabolism and magnesium metabolism are closely related [22]. Along-term high-magnesium diet leads to thyroid dysfunction, whereas hypomagnesemia may lead to a rapid recurrence of GD, and magnesium supplementation can promote the normalization of thyroid morphology and function [23]. AITD is a complex genetic disease, and the genes leading to AITD disease can be divided into two categories: immunomodulatory genes, including human leukocyte antigen (HLA), cytotoxic T lymphocyte-associated antigen 4 (*CTLA-4*), protein tyrosine phosphatases, nonreceptor type 22 (*PTPN22*), CD40, CD25, and Fc receptor-like 3 (*FCRL3*) genes, as well as thyroid-specific genes, including thyroid-stimulating hormone receptor (*TSHR*) and thyroglobulin (*Tg*); however, currently, there is no evidence that any of these genes are associated with *SLC12A3* [20]. Thyroid dysfunction affects kidney physiology and development, and conversely, kidney disease may cause thyroid dysfunction. Hyperthyroidism leads to increased glomerular filtration rates and activation of the renin-angiotensin-aldosterone system [24]. Patients with thyroid disease may experience symptoms of GS [25]. Many kidney diseases such as chronic kidney disease and glomerulonephritis are related to thyroid dysfunction, including reduced serum T3, T4, or Hashimoto's thyroiditis [26–28]. Most GS patients are referred to the endocrinology department, as thyroid dysfunction can lead to hypokalemia and hypomagnesemia. For this reason, compared with healthy people, GS patients receive thyroid function tests more frequently.

As of today (24/04/2021), the Clinvar database contains 444 mutations with clinical significance, including conflicting interpretations (23), benign (51), likely benign (73), uncertain significance (150), likely pathogenic (44), and pathogenic (103). The database also contains frameshift, missense, nonsense, splice site, ncRNA, UTR, and other mutation molecular consequences, of which missense is the most common (https://www.ncbi.nlm.nih.gov/clinvar/?term=SLC12A3). Compound heterozygous mutations are more common than homozygous mutations [6]. Among Chinese GS patients, compound heterozygous mutations accounted for 72.5%, and missense mutations accounted for more than 72% of different mutations in the *SLC12A3* gene [29]. The missense mutation Arg83Gln is more common in the GS pedigree, but the pathogenic mechanism remains unclear [30]. Zeng et al. found that among the 137 cases of GS patients in China, six patients carried compound heterozygotes of Arg83Gln, among which two patients also carried three responsible mutation points [29]. The mutant found in proband A: NC_000016.10:g.56872655_56872667 (gcggacatttttg>accgaaaatttt) is composed of multiple mutations, including NM_001126108.2:c.976delG mutation, which has been confirmed to be pathogenic [31, 32]. Some researchers believe that the NC_000016.10:g.56872655_56872667 (gcggacatttttg>accgaaaatttt) mutation is a deletion of the genomic region containing a part of exon 8 (C.965-1 _ 976 delinsacgaaatttt) of *SLC12A3*, which is expected to destroy RNA splints and possibly lead to the deletion or destruction of protein products. This mutation has been described as “c.965-1 969delGCGGACinsACCGAAA & c.976 977delGT” and “Intron 7 1 G>A & Ex8 nt +1 to +12 delCGGACATTTTTGinsCCGAAAATTTT” [33–35]. Some researchers have suggested that the upregulation of TRPV5/6 and of ROMK1 and Maxi-K are involved in the pathogenesis of hypocalciuria and hypokalemia in NCC Ser707X knockin mice and human GS, respectively [33]. Glaudemans et al. found that the Thr392Ile mutant did not show transport activity, while the Asn442Ser and Gln1030Arg NCC mutants showed reduced NCC plasma membrane localization and therefore a reduced function of NCC, which may relate to an impaired transport function. The experiment also revealed that the transporters could still reach the plasma membrane even if the NaCl absorption of NCC mutants Glu121Asp, Pro751Leu, Ser475Cys, and Tyr489His was blocked, indicating that they affect the ion affinity of NCC [34]. From the study of the deletion function of these mutants, we found that the NC_000016.10:g.56872655_56872667 (gcggacatttttg>accgaaaatttt) mutation can be classified as pathogenic. The mother of proband A alone carried the heterozygous mutation NC_000016.10: g.56872655_56872667 (gcggacatttttg>accgaaaatttt), and according to the recessive inheritance rule, the carrier should be clinically and metabolically asymptomatic, but she had long-term hypokalemia. It was reported that about 18-40% of patients clinically diagnosed with GS carried only one allele mutation in *SLCl2A3*, detected by direct sequencing [30]. Among the 67 Chinese GS patients, the screening also found that 16.4% only carried one mutant allele [36]. The possible reasons for this situation are (1) the mutation site may be located in the unsequenced *SLCl2A3* regulatory fragment, such as the 5′or 3′ untranslated region, promoter and enhancer regions, or intron depth [37]; (2) there may be large-scale gene recombination, involving one or more exons, which are difficult to detect by single exon sequencing [38]; (3) the expression of NCCT cotransporters may be affected by epigenetic modifications and/or silent polymorphism, which interfere with its function [38]; and (4) other pathogenic gene mutations may be related to GS. Zelikovic et al. found that, in addition to *SLC12A3*, the R438H mutation of *CLCNKB* may play a role in the pathogenesis of GS [39]. Among the 137 GS patients in China, 9 patients were found to carry the Arg904Gln mutation, and therefore, these can be regarded as frequent mutations [29]. Arg904Gln may be an area for increased research in Chinese GS patients [36]. Bioinformatics analysis showed that if the wild-type 904Arg was replaced by the mutant allele 904Gln, the three-dimensional structure of the *SLC12A3* protein will change significantly, and the Arg904Gln mutation may have important physiological significance [40]. Tanaka et al. believed that the Arg904Gln gene variation in *SLC12A3* could reduce the risk of diabetic nephropathy in type 2 diabetes mellitus (T2DM) [41]; however, other studies have provided evidence supporting the correlation between Arg904Gln variant and the disease development of diabetic nephropathy in patients with T2DM and GS, suggesting that this variant may be a key predictor of end-stage renal disease [42, 43]. Several suspected pathogenic mutations were found near our newly discovered heterozygous mutant of Asp839Val (c.2516A>T): C.2490C>T (p.Thr830=), c.2495A>G (p.Asp832Gly), c.2532G>A (p.Trp844Ter), c.2510_2511del (p.Leu836_Phe837insTer), c.2514C>T (p.Asp838=), c.2521G>A (p.Gly841Ser), c.2533del (p.Leu845fs), and c.2546T>A (p.Leu849His) (https://www.ncbi.nlm.nih.gov/clinvar). These mutations can lead to protein product deletion or destruction, and we speculate that since Asp839Val is located in this region, it may also be a pathogenic mutation.

Individualized lifelong oral potassium or magnesium supplementation or both are the main methods for the treatment of patients with GS. In the case of hypomagnesemia, magnesium supplementation is the initial treatment, as magnesium supplementation promotes potassium supplementation and reduces the risk of tetany and other complications [44, 45]. The current consensus recommends that the therapeutic targets of serum potassium and magnesium are 3.0 mmol/L and 0.6 mmol/L, respectively [46, 47]. If there is persistent and symptomatic hypokalemia, poor efficacy of the supplements, or an unacceptable level of side effects, other medications can be used, such as potassium-sparing diuretics [48, 49], renin angiotensin system blockers [50], or nonsteroidal anti-inflammatory drugs, such as indomethacin. A combination of both kinds of treatment can also be [51–53] recommended. However, angiotensin-converting enzyme inhibitors (ACEI) and angiotensin receptor blocking (ARB) are not recommended for treating GS due to their increased risk of hypovolemia. The potassium-sparing diuretics amiloride, spironolactone, and eplerenone are all useful for the treatment of GS, as they increase the serum potassium levels in patients resistant to potassium supplementation, and also treat magnesium deficiency worsened by elevated aldosterone levels [48]. Indomethacin is rarely used in GS because plasma prostaglandin E2 (PGE2) levels in GS patients are usually normal. However, some GS patients have significantly higher levels of PGE 2 and PGE 2 metabolites (PGEM) in urine and plasma, while elevated urine PGEM levels indicated severe clinical manifestations, and the COX 2 inhibitor may be a potential therapeutic target in GS patients with increased PGEM [54]. In an open, randomized, crossover study comparing the efficacy and safety of 75 mg indomethacin, 150 mg eplerenone, and 20 mg amiloride in GS patients, each drug increased plasma potassium levels by about 0.3 mmol/L [55]. Although effective against hypokalemia, indomethacin and other nonsteroidal anti-inflammatory drugs should be used cautiously because of their short- and long-term gastrointestinal side effects and nephrotoxicity. It is worth noting that proton pump inhibitors can affect the biological activity of magnesium, thereby reducing its intestinal absorption [56]. Therefore, it is recommended to increase the intake dose of magnesium appropriately if proband A is taking proton pump inhibitors in relation to chronic gastritis.

In summary, *SLCI2A3* test not only helps in the diagnosis and treatment of clinically suspected GS patients but can also be used to screen the family members of patients, to provide for the early detection, prevention, and treatment of the disease. In this study, we found relevant new pathogenic mutations and also found that some GS patients with long-term hypokalemia can contract kidney damage, which has been confirmed by kidney tissue biopsies; however, whether GS patients are susceptible to complicated thyroid disease needs to be confirmed by a large sample of evidence-based research. We also summarized the new advances in GS treatment, hoping to help clinical workers better understand the pathogenesis and physiological processes of the disease.

## 5. Conclusion

It was found that SLC12A3 gene detection contributes to the diagnosis of GS, and the newly discovered SLC12A3 mutation enriches the GS gene mutation spectrum. Chronic GS can cause renal impairment. Whether GS patients are susceptible to complicated thyroid disease needs to be confirmed by a large sample of evidence-based medicine.

## Figures and Tables

**Figure 1:** (a) Family A genetic pedigree map; black indicates a carrier of the Arg83Gln mutation, gray indicates a carrier of the mutation of *SLC12A3* NC_000016.9:g.56872655_56872667 (gcggacatttttg>accgaaaatttt), the arrow indicates the proband, the square indicates male, and the circle indicates female; (b) family B genetic pedigree map; black indicates a carrier of the Asp839Val mutation, gray indicates a carrier of the Arg904Gln mutation, the arrow indicates the proband, the square indicates male, and the circle indicates female; (c–e) pathological electron microscopic examination of renal biopsy shows swelling and vacuolar degeneration of glomerular epithelial cells, diffuse proliferation of mesangial cells and matrix, accompanied by a small amount of low-density electron dense deposition, swelling, and vacuolar degeneration in the visceral epithelial cells, segmental fusion of epithelial cells foot processes. (f–i) Pathological light microscopic examination of renal biopsy shows mild mesangial hyperplasia in the focal segment of the glomerulus, hyperplasia, and hypertrophy of juxtaglomerular apparatus cells, mild renal tubulointerstitial lesions, and one glomerular sclerosis (h). (f) HE staining ×200; (g, h) PAM staining ×200; (i) PAS staining ×200.

**Figure 2:** Sanger sequencing image of Pedigree A mutation type. (a) The NP_001119580.2:p.Arg83Gln (NM_001126108.2:c.248G>A, rs768527231) heterozygous mutant type in *SLC12A3* exon1; (b) the corresponding wild type; (c) the NC_000016.10:g.56872655_56872667 (gcggacatttttg>accgaaaatttt, rs1215667472) heterozygous mutant type in exon8; (d) the clone of the mutant type at the corresponding position; and (e) the clone of the wild type at the corresponding position.

**Figure 3:** Sanger sequencing diagram of Pedigree B mutation type. (a) The Asp839Val (c.2516A>T) heterozygous mutant type in *SLC12A3* exon21; (b) the corresponding wild type; (c) the NP_001119580.2:p.Arg904Gln (NM_001126108.2:c.2711G>A, rs11643718) heterozygous mutant type in exon23; (d) the wild type at the corresponding position.

**Table 1:** The exon primer and PCR condition of *SLC12A3* gene.

Exon	Primer sequence (5′-3′)		Annealing temperature (°C)	Length (bp)
	Forward	Reverse		
1	CTATAAAACCACCCTGTGTGTCCTT	GAAGTGGCCAGTCTTCTGAGAC	55	374
2	CCTCAAGCAGCTCAACACC	GCCTGAGAGTCAGAGCTGAG	55	375
3	TACTGAAGTGGGTGAAGAAGGGA	CTGAGACTGAACCAGGGAGGAGAA	60	372
4	CTCCCAAAGTGACAGAGACCCAT	GGGAGTCCTGTTCCCAGGATTA	55	311
5	CCAACCGACTCATCTGGTTTCA	CACTCTCACCCACAGTGATCAG	55	330
6	AACATCGTCCTAGCAGAGTGC	TCCAGCATGGACATCGAGC	60	372
7	CTTGAACAGATCCTGCTGCATAATG	CCTGACCATGGGATTGGGTAAT	55	375
8	TGGGAGGATGGGATTACCCAAT	GGACTGGACTGGATTTTAGAAGCC	52	372
9	CGACCCGTGATCTTGGTTGTAT	CACTTACCAATGGTGGCTGAGAT	60	329
9	GCCATTTTCTGGACGACCATTT	TCTCCCTGTTGTTAGAGAGTCGAA	60	171
10	GCTGGAAGAGGACAGAGTAAGGA	CTCTCCTAAGCCTAGGCCTCAA	60	344
11	GTAGGGAATGAAGTGCCACAGAT	CCTTCAGGTGTTTGTAGCAGTCA	60	286
12	GCAACTCCACCATTCAAGCTCT	AGCCTTACCGATGATGATGAAGG	55	375
12	AGGCTATGGCAAGAACAAGGAG	CTCTTAGTGCCCACTAACTGTCAG	55	208
13	TCACAGATGAGAAGGTTGAGACTGA	TCAATGGTTTTAAATTGAGAGGTGACCTT	60	368
14	GGGATGTCCTGTGGCTGTATTT	CATGATGACCACGGAGATGATAGC	60	330
14	AGACCTTCATTCCAATACTACAACAAGTG	GCCACATTGGGAGGGATAAAGG	60	303
15	TGCCTAGAGAAGGCCGACATTA	CCATGTCTGTTCCCTCTCTGAGT	60	344
16	GGAAGGACCAGGGAGACTAGTG	ACGTGGCCACAGATCATCAG	60	320
16	GGACTTTGTGGGCACCTTCA	TCTGTGGGTGGACATCACAC	60	230
17	CCCACTCCTTGTGTTTTCCCTTA	GACTTTCTGCCTTCCAGGTTGT	60	363
18	TTTTTGAGAATCAGCACATCTGGAGA	GCCCAGCAGGACTCAACTTTTTA	55	326
19	CCAATTCTGCCTGTACAGGATACA	GGGACCATTAAGAGGCGACTTT	55	375
20	GGGACTTTCTTCCTAGCATTAAGGG	CACCTGTCCTCGACCAAGTT	60	266
21	GAATGGAGAGTGCACTTCCCTA	GTCACTGACCTCCATCGTCAAA	60	372
21	CAGGGCAAGAAGACCATAGACATC	CTCTCAAAGCTTCCCATTTTATAACCAAAA	60	239
22	GCGACTTGAATTCAGTCAGCCAT	GTGGTGGTAGAGGATCTAGGGTA	60	369
23	GGTGCTCAGTGAAAATTAGTTGAATGAAT	CGGAACTTGCTCAGCAGAGAA	60	375
23	TCCATGTGTCCTCCAGGATCAT	CTCCTAGTCTACCAAGGAAAAAGGG	60	198
24	GGGACACAATCTGATTTGTTCACTG	TCATCCTTGAAGCCATCATTCAGAC	55	375
24	CACCAAGAGGTTTGAGGACATGAT	CAAGGATAGCACTGAGTTCCACA	55	329
25	CTTCCTGGAGACAGGAGACTCTAT	CCAGGGCTATGTTTATGGGAACT	60	374
26	GCTCTGAGGGACGGTAAACAGA	GCCACTTAAAGTGCAACAGAACAT	55	362

**Table 2:** Clinical and biochemical characteristics in index cases of GS.

Variable	Proband A	Proband B	Normal value
Blood gas analysis			
PH	7.481	7.460	7.35~7.45
PaCO_2_ (mmHg)	35.2	40.7	35~45
BE (mmol/L)	5.2	5.4	-3.0~+3.0
SB (mmol/L)	29.0	29.2	21.3~24.8
AB (mmol/L)	28.0	29.4	21.4~27.3
Biochemical indexes			
Serum sodium (mmol/L)	138	135	137~147
Serum potassium (mmol/L)	3.2	2.2	3.5~5.3
Serum chloride (mmol/L)	96	92	99~110
Serum calcium (mmol/L)	2.25	2.34	2.11~2.52
Serum magnesium (mmol/L)	0.50	0.38	0.75~1.02
Serum phosphate (mmol/L)	0.87	0.99	0.85~1.51
Blood urea nitrogen (mmol/L)	3.2	5.37	2.1~7.1
Creatinine (mmol/L)	43	54	40~135
GFR (mL/min)^#^	85.8	94.6	80~120
Glucose (mmol/L)	4.62	5.56	3.9~6.1
Renin angiotensin aldosterone system			
Renin activity (*μ*g/L• h) [lie]	12.22	6.34	0.05~0.79
Angiotensin II (ng/L) [lie]	95.99	66.46	28.2~52.2
Aldosterone (ng/L) [lie]	116.73	87.47	59.5~173.9
Corticotropin and cortisol levels			
ACTH (pg/mL) [16 pm.]	17.6	12.6	7.2~63.6
Cortisol (nmol/L) [16 pm.]	165.4	221.8	58~395
Urine tests			
Urine protein	—	++	—
24-hours proteinuria (g/24 h)	0.012	0.823	<0.15
24-hour urine potassium (mmol/day)	33.4	77	25.0~125.0
24-hour urine calcium (mmol/day)	0.2	1.4	2.5~7.5
24-hour urine sodium (mmol/day)	108	335	40~220
24-hour urine chlorine (mmol/day)	115	223	170~255
24-hour urine phosphorus (mmol/day)	6.7	22.2	12.9~42.0
24-hour urine magnesium (mmol/day)	5.5	5.0	3.0~5.0
Urine calcium/creatinine (mmol/mmol)	0.0002	0.001	<0.2
Thyroid function index^∗^			
TSH (mIU/L)	6.19	0.94	0.27~4.2
TPOAb (IU/mL)	>600.00	7.17	0~34
FT3 (pmol/L)	4.80	5.70	3.1~6.8
FT4 (pmol/L)	14.24	18.03	12~22
TGAb (IU/mL)	740.00	<10.00	0.1~115

^#^GFR by MDRD clearance (mL/min); ^∗^thyroid function index of the older sister of proband B: TSH 0.10 mIU/L, TPOAb 341.10 IU/mL, FT3 5.04 pmol/L, FT4 18.93 pmol/L, TGAb 545.40 IU/mL (normal value as above).

**Table 3:** Summary on 2 pedigrees with GS family with SCL12A3 gene (Nm_001126108.2) mutant genotype.

	Nucleotide change	Mutation	Predicted effect	Exon	Number in dbSNP
Pedigree A					
II5,6	c.248G>A	p.Arg83Gln	Het, missense	1	rs768527231
	NC_000016.10:g.56872655_56872667 (gcggacatttttg>accgaaaatttt)		Het, splice site/frame shift	8	
II4	C.248G>A	p.Arg83Gln	Het, missense	1	rs768527231
I2; II1, 3; III1, 2	NC_000016.10:g.56872655_56872667 (gcggacatttttg>accgaaaatttt)		Het, splice site/frame shift	8	
Pedigree B					
II2, 3	c.2516A>T	p.Asp839Val	Het, missense	21	
	c.2711G>A	p.Arg904Gln	Het, missense	23	rs11643718
I1; III1, 2	c.2516A>T	p.Asp839Val	Het, missense	21	
I2; III3	c.2711G>A	p.Arg904Gln	Het, missense	23	rs11643718

Het: heterozygous mutation.

## Data Availability

The datasets used and/or analyzed during the present study are available from the corresponding author upon reasonable request.
